RETRACTED

# Effects of GABAB receptor activation on spatial cognitive function and hippocampal neurones in rat models of type 2 diabetes mellitus

**DOI:** 10.1042/BSR20171184

**Published:** 2018-01-19

**Authors:** Xiao-Jun Cai, Lei Wang, Chun-Mei Hu

**Affiliations:** 1 Heilongjiang Academy of Traditional Chinese Medicine, Harbin 150036, P.R. China; 2 The Third Hospital of Heilongjiang, Beian 164000, P.R. China

**Keywords:** Gamma-aminobutyric acid type B, Hippocampal neurons, Rat models, Spatial cognitive function, Type 2 diabetes mellitus

## Abstract

The present study was conducted with the aim being to investigate the effect γ-aminobutyric acid type B (GABAB) receptor activation have on spatial cognitive function and hippocampal neurones found in the rat models of type 2 diabetes mellitus (T2DM). T2DM rat models were then established, randomized, and subsequently assigned into normal control (NC), T2DM, T2DM + chemical grade propylene (CGP), T2DM + baclofen, and T2DM + CGP + baclofen groups. T2DM rats’ weight and blood sugar concentrations were monitored. The DMS-2 Morris water maze testing system was performed in order to figure out the spatial cognitive function of these rats. Reverse-transcription quantitative PCR (RT-qPCR) and Western blotting were also performed in order to detect *GABAB* mRNA and protein expressions. We used the Nissl staining method in order to detect the number of hippocampal neurones, TUNEL (terminal deoxyribonucleotidy transferase-mediated dUTP nick labeling) staining to detect cell apoptosis, and Western blotting method in order to measure the expressions of the apoptosis-related proteins (Bax, cytochrome *c* (Cyt-*c*), Caspase-3, and Bcl-2). In comparison with the T2DM group, the weight decreased, blood sugar concentration increased, and spatial cognitive function as well as hippocampal neurones were both impaired in the T2DM + CGP group, contrary to the rats in the T2DM + baclofen group who showed an opposite trend. The situation in the T2DM + CGP + baclofen group was better than that found in the T2DM + CGP group while proving to be more serious than that of the NC and T2DM + baclofen groups. Conclusively, activating the GABAB receptor improved spatial cognitive function and hippocampal neurones in the T2DM rats.

## Introduction

Type 2 diabetes mellitus (T2DM), a complicated chronic metabolic disease, demonstrates a heterogeneous etiology with serious complications [1]. T2DM is featured by hyperglycemia with the majority of patients being elderly [2]. In 2014, approximately 387 million people were patients diagnosed with diabetes worldwide and its prevalence is estimated to reach approximately 592 million patients diagnosed with diabetes by year 2035 [3]. As a significant obstacle to the world’s healthcare system, T2DM has become prevalent worldwide, especially in Asia where over 60% of patients are affected by T2DM [4]. The major cause of the prevalence of T2DM amongst the human population happens to be genetic factors, while other factors like obesity, rapid urbanization, and lack of exercise also play critical roles in the rapid increased expansion of T2DM [5]. Patients affected by diabetes show a higher possibility of cognitive deficits, which show influence predominantly on the areas of attention, psychomotor efficiency, learning and memory, executive function, mental flexibility, and speed, as well as an increased risk of developing various dementia [6]. Therefore, it is significantly important to explore an effective way to treat T2DM and recently gene therapy has been popularly used in treating T2DM.

γ-Aminobutyric acid type B (GABAB) receptors are heterodimeric G-protein-coupled receptors (GPCRs), which are made up of GABAB1 and GABAB2 subunits [7]. GABAB receptors play an important part in regulating a lot of synapses including the pre- and post-synapses and are regarded as some of the most interesting targets for the treatment of numerous brain diseases, including addiction [8]. Furthermore, it is recognized that GABAB receptors are significant in regulating circuit excitability throughout the brain by directly affecting different postsynaptic glutamate receptors, that is, GABAB receptors have an influence on the activity and signaling of glutamate receptors both physiologically and pathologically [9]. In addition, according to a relevant research, there were certain occurrences involving significant alterations of the GABAB receptor density and functionality between several brain regions related to cognitive functions such as hippocampus, which would suggest that to some extent, spatial learning and memory may be associated with GABAB receptors [10]. As a result, it can be speculated that the GABAB receptors may be related to both spatial cognitive function and hippocampal neurones. In association with these findings, the present study is aiming to investigate the effect of the activation of the GABAB receptor on spatial cognitive function and hippocampal neurones in the rat models of T2DM.

RETRACTED

## Materials and methods

### Ethics statement

The present study was performed in co-operation with the approved animal protocols and guidelines established by the Medicine Ethics Review Committee for animal experiments (number 201506003). All experiments were in strict agreement with relevant regulations set by the International Association for the Study of Pain for the protection and use of laboratory animals [11].

### Experimental animals

A total of 60 healthy male Sprague–Dawley (SD) rats (age: 4-month-old; weight: 200–250 g) at clean grade were chosen to take part in the present study. All rats were purchased from SLRC Laboratory Animal Company, Shanghai, China and raised at room temperature, between 21 and 23°C. The clean grade animal facility had a constant humidity of 60% ± 5% with good ventilation. The rats were raised in a quiet environment with a normal circadian rhythm while being provided with sufficient drink and food nourishment.

### Model establishment and animal grouping

The weight of the rats was measured using a BSA223S-CW (Mettler Toledo, Shanghai, China) and the blood was collected after location of the tail vein before beginning the experiment. Ten SD rats were chosen as part of the normal control (NC) group with conventional feeding. The remaining 50 rats were fed a high-glucose and high-fat diet containing 20% sucrose, 0.25% pig bile salt, 10% lard, 2.5% cholesterol, and 67.25% normal feed (Botai Biotechnology Co., Ltd., Beijing, China). After 1 month, 50 rats were intraperitoneally injected with streptozotocin (STZ; Sigma–Aldrich Chemical Company, St. Louis, MO, U.S.A.) at 35 mg/kg, which was then dissolved in 0.1 mmol/l citrate buffer solution (pH 4.4). The 50 rats were then treated with normal feed. The NC group was injected with an equal amount of citrate buffer solution. Two weeks after injection of STZ, blood was collected from the 50 rats in their tail vein in order to measure random blood sugar. If either the concentrations of random blood sugar were above or equal to 16.7 mmol/l, the model was regarded as being successfully established [12]. To this discoveries’ discredit, three unsuccessful rat models were excluded. The rest 47 successful rat models were randomly selected and assigned to four groups (ten rats in each group): T2DM group, T2DM + chemical grade propylene (CGP) group, T2DM + baclofen group, and T2DM + CGP + baclofen group. The treatment regimens of each group are shown in Table 1. The rats were weighted and their tail vein blood was collected soon after. Baclofen (Sigma–Aldrich Chemical Company, St. Louis, MO, U.S.A.), acting as the GABAB receptor agonist, was given to rats by an intraperitoneal injection at expressions of 5 mg/kg every day. CGP 55845 (Tocris Bioscience, Bristol, England), acting as the GABAB receptor blocker, was given to rats by intraperitoneal injection at expressions of 1 mg/kg every day. After grouping, the rats were then treated consecutively for 1 week with a medication intervention. At 0.5 h after each injection, behavioral tests were conducted on the rats.

RETRACTED

**Table 1:** Treatment regimens for the rats in each group

Group	Treatment regimen
NC group	Normal rats treated with normal saline
T2DM group	T2DM rats treated with normal saline
T2DM + baclofen group	T2DM rats treated with 5 mg/kg/day baclofen
T2DM + CGP group	T2DM rats treated with 1 mg/kg/day CGP 55845
T2DM + CGP + baclofen group	T2DM rats treated with 1 mg/kg/day CGP 55845 and 5 mg/kg/day baclofen

### Behavioral testing

A behavioral testing was performed using the DMS-2 Morris water maze testing system (RWD Life Science, Shenzhen, China). The system consisted of a rat’s behavior test system, an image acquisition system, and a computer data processing and analysis system. The Morris water maze is a black cylindrical tank (0.5 m in height and 1.2 m in diameter) with a constant temperature heating device installed at the bottom. There were no landmarks found in the water maze, and a camera was set above the maze. During these tests, the environment was kept quiet to block out any interference, and the temperature was maintained between 22 and 25°C. The place navigation test was carried out and the resulting escape latency was used for measurement index purposes. The water area was divided into four quadrants of equal size and the rats facing the wall of the tank were put into one of the quadrants at random selection. If a rat found its way to the platform within 60 s and remained on the platform for 5 s, the duration of its swimming was recorded as its escape latency. If a rat could not find its way toward the platform in 60 s, the rat was then guided to the platform and remained there for 15 s, with the escape latency recorded as 60 s. These experimental procedures were repeated multiple times and the average value was subsequently calculated. The spatial probe test was conducted. The swimming time in the target quadrant was then recorded. The platform was then removed and the rats facing the wall of the tank were then put into the target quadrant. During the following 60 s, the swimming time of the rat was observed, and the residence time(s) when the rat was still in the original quadrant was calculated. The tests started when the rats were treated and ended until the finish of the treatment, altogether 7 days.

### Measurement of blood sugar concentration

Blood obtained from the rat’s tail vein before the experiment, treatment, and death was all preserved. Working fluids were prepared according to the instructions provided by the Hoffmann-La Roche AG Kit (Basel, Switzerland) and were then added in with the sample or the standard according to the instructions. After mixing, the reaction was observed for 10 min at a temperature of 37°C. An ultraviolet-visible spectrophotometer (Thermo Fisher Scientific, California, U.S.A.) was used in order to measure the optical density (OD) of each tube calibrated at 500 nm operating wavelength and 1 cm optical path. The glucose concentration (mmol/l) of each group was calculated as such: glucose concentration = standard concentration × [OD_(sample)_ − OD_(blank)_]/[OD_(standard)_ − OD_(blank)_].

RETRACTED

### Sample collection

After behavioral tests concluded, rats amongst the five groups were kept hydrated and fed for 2 days. The rats inhaled 3% isoflurane (Jiangsu Hengrui Medicine, Co., Ltd., Lianyungang, China) for 1 min in order to experience deep anesthesia. Short-time isoflurane anesthesia does not affect hippocampal or biochemical functions. The rat limbs were then immobilized and their chest cavities were quickly opened in order to expose their cardiovascular region. A 16G venous puncture needle (B. Braun Melsungen AG, Melsungen, Germany) was inserted into the aorta by puncturing a hole through the left ventricle. The auricula dextra was then cut and quickly infused with a 200 ml cold saline solution. The rats’ bodies were no longer of use for this experiment and were rapidly executed with removal of their brains following soon after. The brain tissues were quickly transferred on to ice made from double distilled water in order for preservation. The hippocampal tissues were then quickly isolated, rinsed with 4°C sterile water, dried, and placed in liquid nitrogen before frozen in a freezer under −80°C conditions. The hippocampal tissues were ultimately used for tissue sections and were anesthetized and rapidly perfused with a heparinized saline (Boster Biotechnology Co., Ltd., Wuhan, China), finally being fixed with 200 ml of 4% polyformaldehyde (Boster Biotechnology Co., Ltd., Wuhan, China).

### Reverse-transcription quantitative PCR

The total RNA in the cryopreserved hippocampal tissues was extracted by using TRIzol (Invitrogen Inc., Carlsbad, CA, U.S.A.) according to the instructions provided by the kit. The RNA purity and concentration expressions were measured using a NanoDrop 2000 spectrophotometer (Thermo Fisher Scientific, CA, U.S.A.). The PCR primers were designed using the Premier 5.0 software in co-operation with the gene sequences published in the GenBank database and were subsequently synthesized by the Shanghai Sangon Biological Engineering Technology & Services Co., Ltd., Shanghai, China. The PCR primers are listed in Table 2. The PCR was performed using an ABI PRISM 7500 qRT-PCR System (ABI, Carlsbad, CA, U.S.A.). The reaction system was prepared according to the instructions provided by the One Step SYBR® PrimeScript® PLUS RT-PCR Kit (Takara Biotechnology Ltd., Dalian, China). PCR conditions were predenaturation at temperatures 95°C for a 5-min period, 40 cycles of 95°C denaturation for 30 s, 61°C annealing for 30 s, 72°C extension for 1 min, and finally extension at 72°C for a total of 5 min. Glyceraldehyde-3-phosphate dehydrogenase (GAPDH) was used as the internal reference for this portion of the experiment. Each gene provided in the samples was measured in triplicates. The reliability of the PCR results was confirmed by using the dissolution curve with the cycle threshold (*C*_t_) value. The relative gene expression was calculated using the 2^−ΔΔ*C*^_t_ method [13]: Δ*C*_t_ =*C*_t__(target gene)_ − *C*_t(internal reference)_, ΔΔ*C*_t_ =Δ*C*_t(experiment group)_ − Δ*C*_t(control group)_.

RETRACTED

**Table 2:** Primer sequences for reverse-transcription quantitative PCR

Gene	Sequence
*GABAB*	Forward: 5′-AGCTGACCAGACCTTGGTCATT-3′
	Reverse: 5′-AACTGGCTTCTCCCTATGTGG-3′
*GAPDH*	Forward: 5′-GATGGGTGTGAACCACGAGAAAT-3′
	Reverse: 5′-ACGGATACATTGGGGGTAGGAA-3′

### Western blotting

The total proteins found in the cryopreserved hippocampal tissues were extracted using TRIzol (Invitrogen, Waltham, MA, U.S.A.) according to the instructions provided. The protein concentrations were measured using a BCA Kit (Beyotime Biotechnology, Shanghai, China). The extracted proteins were then added in with a buffer solution and boiled for a total of 10 min at a temperature of 100°C. The proteins were then separated using the 10% PAGE (Boster Biotechnology Co., Ltd., Wuhan, China). During use of PAGE, each well was added with approximately 30 µg of samples, and the electrophoresis voltage was calculated at 60 V in a concentrated gel for 45 min, and then in separation gel for 1 h at 120 V. The membrane applied was PVDF. The protein was transferred with a constant current of 250 mA for 2 h. Then, the extracted proteins were blocked at room temperature in 5% BSA for 1 h, and incubated with the primary antibodies GABAB (ab55051), Bax (ab32503), Cyt-*c* (ab104342), Bcl-2 (ab32124), Caspases-3 (ab2171), and β-actin (ab8226) (all 1:1000; Abcam Inc., Cambridge, MA, U.S.A) overnight at a temperature of 4°C. The samples were rinsed a total of three times (each 5 min) using a TBS and Tween 20 (TBST) solutions. Next, the samples were incubated with the corresponding second antibodies at room temperature for 1 h. The samples were also rinsed a total of three times using the TBST solutions (5 min each time). The samples were developed using ECL chemiluminescence reagent (Beyotime Biotechnology, Shanghai, China), and the gray values of the target bands were analyzed using the ImageJ software.

### Nissl staining

Paraffin-embedded hippocampal tissue was sectioned at a thickness of 4 μm. The sections were immersed in xylene I and II solutions, respectively for 30 min. After washing with 100%~70% gradient alcohol (each for 10 min), the sections were then washed twice with double distilled water and stained for 20 min with 0.5% Nissl staining solution. The sections were then washed with double distilled water once more, this time rapidly, color-separated by using a 95% hydrochloric acid alcohol for 1 s and dehydrated using the gradient alcohols and xylene. The sections were then sealed with a neutral balata. All reagents were acquired and purchased from Boster Biotechnology Co., Ltd., Wuhan, China. An Olympus microscope was used in order to observe the sections. At low magnification, three grid visual fields (CA1 area, CA3 area, and DG area) of each side of the hippocampus were selected and took part as the sampling area in each hippocampal slice. The number of cells with an intact membrane, plump nuclei, and clear nucleoli in the CA1, CA3, and DG regions of hippocampus in the same field was counted using 25 μm^2^ counting plate in high power filed (×40), with the ImageJ software being used for counting and analysis. This experiment was repeated three times.

RETRACTED

### TUNEL staining

A TUNEL (terminal deoxynucleotidyl transferase-mediated biotinylated dUTP nick end labeling) staining was implemented in order to detect cell apoptosis in hippocampal neurones. Frozen sections were then prepared from fresh hippocampal tissue, dried at room temperature, and ultimately sealed in a 3% BSA Tris/HCl (Roche, Basel, Switzerland) for 1 h. A nonspecific reaction was blocked. The sections were then washed with PBS and incubated for 1 h at a temperature of 37°C with an addition of 50 μl of TUNEL reaction mixture. The endogenous peroxidase was blocked using 3% H_2_O_2._ The sections were then incubated for 30 min with a peroxidase-labeled fluorescent antibody, followed by three washes with PBS. After glycerol mounting, the sections were observed under an Olympus fluorescence microscope. Each section of the hippocampal area in each rat group was selected. Three loci identified on each side of the hippocampus were observed with TUNEL staining. Three fields were chosen in each section, and subsequently counted and analyzed using the ImageJ software. The cell apoptosis rate was calculated as the ratio of the number of apoptotic cells to that of total cells. This experiment was repeated three times.

### Statistical analysis

All data recorded in the present study were analyzed using the SPSS 18.0 (IBM Corporation, New York, U.S.A.). The measurement data were presented using the mean ± S.D. The goodness-of-fit test was performed for normal distribution. The comparisons between two groups abiding by the normal distributions were analyzed using the *t* test and the comparisons amongst multiple groups were conducted by way of the one-factor ANOVA. *P*<0.05 was identified as having statistical significance.

RETRACTED

## Results

### GABAB expression in rat hippocampal tissues amongst five groups

In comparison with the NC group, the GABAB receptor expression significantly decreased in the T2DM, T2DM + CGP, and T2DM + CGP + baclofen groups (all *P*<0.05). In comparison with the T2DM group, the GABAB expression in the T2DM + CGP group had significantly decreased while there was an increase shown in the T2DM + baclofen group (both *P*<0.05), while no significant difference in GABAB expression was found in the NC group (*P*>0.05). The GABAB expression in the T2DM + CGP + baclofen group was also found to be significantly decreased in comparison with that of the T2DM + baclofen group while simultaneously significantly increased in comparison with that of the T2DM + CGP group (both *P*<0.05), while showing no significant difference when compared with the T2DM group (*P*>0.05) (Figure 1).

**Figure 1:** GABAB expression in rat hippocampal tissues amongst five groups (**A**) *GABAB* mRNA expression in rat hippocampal tissues amongst five groups detected by reverse-transcription quantitative PCR (RT-qPCR). (**B**) Western blotting images of GABAB protein expression in rat hippocampal tissues amongst five groups. (**C**) The gray value of GABAB protein expression in rat hippocampal tissues amongst five groups. *, compared with the NC group, *P*<0.05; ^#^, compared with the T2DM group, *P*<0.05; ^&^, compared with the T2DM + CGP group, *P*<0.05; ^$^, compared with the T2DM + baclofen group, *P*<0.05.

### Weight and blood sugar concentration of the rats amongst five groups

Before the experiment began, the weight and blood sugar concentration of the rats in each group had no obvious difference (all *P*>0.05). Before the treatment, in comparison with that of the NC group, weight had decreased while blood sugar concentration increased in the T2DM, T2DM + CGP, T2DM + baclofen, and T2DM + CGP + baclofen groups (all *P*<0.05). Before execution of rats, in comparison with the NC group, the weight of the rat had decreased while the blood sugar increased in the T2DM, T2DM + CGP, and T2DM + CGP + baclofen groups (all *P*<0.05). In addition, the T2DM + CGP group had shown to have a significant decrease in weight and significant increase in blood sugar concentration, while the T2DM + baclofen group had shown significantly increased weight as well as significantly decreased blood sugar concentration when compared with that of the T2DM group (all *P*<0.05) (Table 3). Therefore, according to the findings listed above, the GABAB receptor agonist baclofen could significantly increase weight while simultaneously showing a significant decrease in blood sugar concentration in the rat models affected by T2DM. GABAB receptor blocker CGP could also significantly decrease weight while significantly increase blood sugar concentration.

RETRACTED

**Table 3:** Comparisons of weight and blood sugar concentration of the rats in each group

Group	Weight (g)			Blood sugar concentration (mmol/l)		
	Before experiment	Before treatment	Before death	Before experiment	Before treatment	Before death
NC group	235.0 ± 9.0	301.3 ± 10.1	320.9 ± 13.1	5.7 ± 1.0	5.4 ± 1.0	4.9 ± 1.1
T2DM group	237.1 ± 7.5	231.0 ± 9.8*	218.7 ± 10.1*	5.8 ± 0.9	25.7 ± 3.1*	31.6 ± 4.1*
T2DM + CGP group	236.5 ± 8.2	233.0 ± 9.8*	201.7 ± 9.7*^†^	5.6 ± 0.8	25.2 ± 2.8*	41.5 ± 4.1*^†^
T2DM + baclofen group	231.7 ± 9.7	227.5 ± 11.1*	317.2 ± 10.7^†^	5.4 ± 0.9	24.9 ± 2.9*	6.5 ± 1.2^†^
T2DM + CGP + baclofen group	238.0 ± 7.3	232.0 ± 9.8*	224.7 ± 10.1^*‡§^	5.6 ± 0.9	24.8 ± 3.1*	29.6 ± 4.1^*‡§^

*, compared with the NC group, *P*<0.05; ^†^, compared with the T2DM group, *P*<0.05; ^‡^, compared with the T2DM + CGP group, *P*<0.05; ^§^, compared with the T2DM + baclofen group, *P*<0.05.

### Escape latency and residence time of rats amongst five groups

In comparison with the NC group, the escape latency was found to have significantly increased, meanwhile the residence time in the original quadrant significantly decreased in the T2DM, T2DM + CGP, and T2DM + CGP + baclofen groups (all *P*<0.05). The difference became increasingly obvious with the extension of the drug intervention time (all *P*<0.05). As previously compared with the T2DM group, the T2DM + CGP group had shown significantly increased escape latency as well as a significantly decreased residence time in the original quadrant. However, the T2DM + baclofen group had shown significantly decreased escape latency and significantly increased residence time in the original quadrant (all *P*<0.05). The difference became increasingly obvious with the extension of drug intervention time (all *P*<0.05). The escape latency found in the T2DM + CGP + baclofen group significantly decreased while in comparison with that of the T2DM + CGP group and also having significantly increased in comparison with the T2DM + baclofen group (both *P*<0.05). The residence time allotted in the original quadrant in the T2DM + CGP + baclofen group had significantly increased in comparison with the T2DM + CGP group while significantly decreased in comparison with the T2DM + baclofen group (both *P*<0.05). With the extension of drug intervention time, the escape latency in the NC and T2DM + baclofen groups both decreased gradually while the residence time in the original quadrant in relation to these two groups increased gradually (all *P*<0.05). Also with the extension of the drug intervention time, the escape latency found in the T2DM + CGP group increased gradually, while the residence time in the original quadrant decreased gradually (all *P*<0.05) (Figure 2). These results subsequently indicated that the activation of the GABAB receptor could drastically improve spatial memory in the rat models of T2DM.

RETRACTED

**Figure 2:** Behavioral testing results for rats among the five groups detected by Morris water maze test. (**A**) Escape latency of rats among five groups. (**B**) Residence time in the original platform quadrant of rats among five groups. *, compared with the NC group, *P*<0.05; #, compared with the T2DM GROUP, *P*<0.05; &, compared with the T2DM + CGP group, *P*<0.05; $ compared with the T2DM+baclofen group, *P*<0.05; NC, normal control. T2DM, type 2 diabetes mellitus, CGP, chemical grade propylene.

### Structure and number of hippocampal neurones in the CA1, CA3, and DG regions in rats amongst five groups

In the NC group, hippocampal neurones had fine structure. A large number of neuronal cell bodies gathered. Nissl bodies appeared as granulate and evenly scattered in the cytoplasm with the nuclei being large round and light in color. In the T2DM group, hippocampal neurones appeared irregularly shaped and the number of hippocampal neurones significantly decreased, the CA3 area became thin, hippocampal neurones were mostly incomplete with an unclear contour of cell bodies in comparison with the NC group (*P*<0.05). The T2DM + CGP group had more of an irregular structure of hippocampal neurones and significantly decreased number of hippocampal neurones in comparison with the NC and T2DM groups (both *P*<0.05). The T2DM + baclofen group had a complete structure of the hippocampal neurones with regular shape and a large number of hippocampal neurones, having no significant difference in comparison with the NC group (*P*>0.05), while having a significant difference in comparison with the T2DM group (*P*<0.05). The T2DM + CGP + baclofen group had an incomplete structure of hippocampal neurones and with the structure being incomplete, a drastically decreased number of hippocampal neurones in comparison with both the NC and T2DM + baclofen groups (*P*<0.05), however having a significantly complete structure and significantly increased number of hippocampal neurones in comparison with the T2DM + CGP group (*P*<0.05) (Figure 3). The aforementioned results indicated that activation of the GABAB receptor could potentially promote the recovery of damaged hippocampal neurones.

RETRACTED

**Figure 3:** Structure and number of hippocampal neurones in rats amongst five groups (**A**) Nissl staining of hippocampal neurones in rats amongst five groups. (**B**) Number of hippocampal neurones in rats amongst five groups; *, compared with the NC group, *P*<0.05; ^#^, compared with the T2DM group, *P*<0.05; ^&^, compared with the T2DM + CGP group, *P*<0.05; ^$^, compared with the T2DM + baclofen group, *P*<0.05.

### Cell apoptosis of hippocampal tissues in rats amongst five groups

No cell apoptosis of the hippocampal tissues found in the NC group. In comparison with the NC group, the cell apoptosis rate in the T2DM, T2DM + CGP, and T2DM + CGP + baclofen groups significantly increased (all *P*<0.05), while showing no significant difference in the T2DM + baclofen group (*P*>0.05). As previously compared with the T2DM group, the cell apoptosis rate significantly increased in the T2DM + CGP group, but decreased in the T2DM + baclofen group (both *P*<0.05). Cell apoptosis rate in the T2DM + CGP + baclofen group significantly decreased in comparison with the T2DM + CGP group while significantly increased in comparison with the T2DM + baclofen group (both *P*<0.05) (Figure 4). Judging by these results, there is significant indication that activating the GABAB receptor could inhibit cell apoptosis.

**Figure 4:** Cell apoptosis of hippocampal tissues in rats amongst five groups (**A**) Cell apoptosis of hippocampal tissues in rats amongst five groups detected by TUNEL staining. (**B**) Cell apoptosis rate amongst five groups; *, compared with the NC group, *P*<0.05; ^#^, compared with the T2DM group, *P*<0.05; ^&^, compared with the T2DM + CGP group, *P*<0.05; ^$^, compared with the T2DM + baclofen group, *P*<0.05. Abbreviation: TUNEL, terminal-deoxynucleotidyl transferase mediated nick end labeling.

### Expressions of apoptosis-related proteins in the rat hippocampus amongst five groups

In comparison with the NC group, the T2DM, T2DM + CGP, and T2DM + CGP + baclofen groups showed higher Bax, Cyt-*c*, and Caspase-3 expressions but a lower Bcl-2 expression (all *P*<0.05). In comparison with the T2DM group, the expressions of Bax, Cyt-*c*, and Caspase-3 all had significantly increased, while the Bcl-2 expression significantly decreased in the T2DM + CGP group (all *P*<0.05). The expressions of Bax, Cyt-*c*, and Caspase-3 were found to have been significantly decreased while the Bcl-2 expression significantly increased in the T2DM + baclofen group (all *P*<0.05). Collaterally, the expressions of Bax, Cyt-*c*, and Caspase-3 in the T2DM + CGP + baclofen group significantly decreased in comparison with the T2DM + CGP group while being significantly increased in comparison with the T2DM + baclofen group (all *P*<0.05). The Bcl-2 expression in the T2DM + CGP + baclofen group significantly increased in comparison with that of the T2DM + CGP group while significantly decreased in comparison with the T2DM + baclofen group (all *P*<0.05) (Figure 5).

RETRACTED

**Figure 5:** Expressions of apoptosis-related proteins in the rat hippocampus amongst five groups (**A**) Western blotting images for expressions of Bax, Cyt-*c*, Bcl-2, and Caspase-3 proteins in the rat hippocampus amongst five groups. (**B**) The gray values of expressions of Bax, Cyt-*c*, Bcl-2, and Caspase-3 proteins in the rat hippocampus amongst five groups; *, compared with the NC group, *P*<0.05; ^#^, compared with the T2DM group, *P*<0.05; ^&^, compared with the T2DM + CGP group, *P*<0.05; ^$^, compared with the T2DM + baclofen group, *P*<0.05.

## Discussion

During the present study, we studied the effects of activating GABAB receptor on spatial cognitive function and hippocampal neurones in rat models of T2DM. Our experimental results showed that the activation of the GABAB receptor had a positive effect on increasing weight, improving spatial cognitive function, promoting recovery of damaged hippocampal neurones, as well as decreasing blood sugar concentration in rat models of T2DM.

According to our results, both the GABAB expression and weight of T2DM rats notably decreased while blood sugar concentration significantly increased. Baclofen significantly increased GABAB expression and weight as well as providing evidence of notable decrease in blood sugar concentration. Decreased weight is directly related to an impaired survival rate in patients with chronic cardiovascular diseases, which are notable risk factors of T2DM [14]. In accordance with the present study, weight loss was often observed in T2DM rats and fasting blood sugar concentration was found in those without diabetes [15,16]. Since maintaining blood sugar concentration within a relatively narrow range is important for the survival of the organism, regulating glycemia as close as possible to a nondiabetic range is the foremost aim in the medical treatment of patients with T2DM and is now achieved clinically primarily through means of suppressing hepatic glucose production [17]. A previous study proved that GABAA channel subunits, α1, α2, β2, and β3, decreased in islets from people with T2DM [18]. Moreover, it was found that activation of the GABAB receptor by baclofen alleviates diabetic neuropathic pain [19]. It was suggested that treatment with baclofen plays a positive role in restraining various alcohol-related behaviors, potentially providing the possibility of the treatment of T2DM [20].

RETRACTED

The present study also proved that the escape latency of rats with T2DM increased while residence time in the original platform quadrant decreased. Activation of the GABAB receptor was also found to have improved spatial memory in rat models of T2DM. A former study indicated that the diabetic rats had significantly increased escape latency as well as a decreased average swimming time in the target quadrant in comparison with that of the control group [21]. Proving consistent with our results, a recent report revealed that T2DM was directly related to impairment of the cognitive function and cognitive impairment had an influence on one-fifth of the patients affected by T2DM at age 60 years or younger [22]. At the present time, it is believed that GABAB1a plays a role in the maintenance of memory and protection from an anhedonic phenotype, while GABAB1b seems to be related to memory formation and potentially developing an anhedonic phenotype [23]. Moreover, GABAB receptor agonist baclofen could also improve the repeated methamphetamine-induced cognitive impairment [24]. GABA is a major inhibitory neurotransmitter in the central nervous system acting at both ionotropic (GABAA and GABAC) and metabotropic (GABAB) receptors [25]. Numerous GABAergic neurones are located in the DG region, and both the GABAA and GABAB receptors in DG regulate synaptic plasticity, learning, and memory processes [26]. Recent studies have indicated that the GABAB receptor blockade suppresses long-term potentiation (LTP) in the DG and impairs spatial learning in the water maze task while GABAB receptor antagonist improved learning and memory formation [27,28].

In addition, our results found that the hippocampal neurones of rats with T2DM were impaired as well as the expressions of Bax, Cyt-*c*, and Caspase-3 were notably increased while Bcl-2 expression notably decreased. Activating GABAB receptor could possibly promote the recovery of hippocampal neurones and inhibit cell apoptosis. A study conducted by Hasnan et al. [29] also showed that Bcl-2 expression was obviously increased in the control group while Bax expression notably increased in the diabetic group. Another previous research also reported that Caspase-3 activation in type 2 diabetic erythrocytes was notably higher than in the control group [30]. It is suggested that increased cholinesterase induced by activating GABAB receptor plays a part in neuronal maturation and stabilization [31]. Some results showed that activating GABAB receptor could notably inhibit oxidative stress-related B-cell apoptosis, and furthermore treatment with GABAB receptor specific agonist may inhibit human B-cell apoptosis [32]. Therefore, it is also assumed that GABAB receptor is a putative target for the improvement of hippocampal neurones and subsequent inhibition of cell apoptosis.

RETRACTED

Thus in our conclusion, the present study provided many compelling evidence that activating GABAB receptor could increase the weight, improve spatial cognitive function, promote recovery of hippocampal neurones, and lower blood sugar concentration in rat models of T2DM. Therefore, the activation of the GABAB receptor may be a potential therapeutic target to treat T2DM. However, many limitations still exist in the present study. The results from this experiment lacked support from relevant clinical data, so the conclusions and results drawn from the present study may not be adequately applied for the general population. Therefore, future studies will be implemented in order to improve our current limitation.

## Abbreviations

CGP: chemical grade propylene
*C*_t_: cycle threshold
GABAB: γ-aminobutyric acid type B
NC: normal control
OD: optical density
SD: Sprague–Dawley
STZ: streptozotocin
TBST: TBS and Tween 20
TUNEL: terminal deoxynucleotidyl transferase-mediated biotinylated dUTP nick end labeling
T2DM: type 2 diabetes mellitus
